# Relationship between Activities of Daily Living of Home-Based Rehabilitation Users and Caregiver Burden-Induced Depression: A Retrospective Study

**DOI:** 10.1155/2022/4524985

**Published:** 2022-06-17

**Authors:** Takuro Ohashi, Takaaki Fujita, Yui Togashi, Yuji Ohashi, Yuta Kisara, Ryohei Jinbo, Ryuichi Kasahara, Yuichi Yamamoto

**Affiliations:** ^1^Department of Rehabilitation, Kita-Fukushima Medical Center, 960-0502, Japan; ^2^Department of Occupational Therapy, School of Health Sciences, Fukushima Medical University, 960-8516, Japan; ^3^Hobara Regional Comprehensive Support Center, 960-0665, Japan; ^4^Yanagawa Hospital, 960-0776, Japan

## Abstract

This study was aimed at determining the cutoff values of activities of daily living (ADL) and the combination of related factors associated with high caregiver burden that induces depression among caregivers. The study participants included 50 pairs of home-based rehabilitation users and their primary caregivers. They were classified into two groups: high-burden and low-burden groups according to the short version of the Japanese version of the Zarit Caregiver Burden Interview score of ≥13 or ≤12, respectively. The cutoff values of ADL and the combination of related factors associated with high caregiver burden were examined using the receiver operating characteristic curve and decision tree analyses. The cutoff value associated with high caregiver burden was 5 points for the controlling bladder item of the Barthel index (BI) (sensitivity: 90%, specificity: 70%). Regarding the decision tree, the controlling bladder item of BI (≤5 or 10 points) was selected as the first layer and the recipient's age (≤78 or ≥79 years) as the second layer. High caregiver burden was identified in 85.7% of the caregivers in whom the score of controlling bladder of BI was ≤5 points and the patient was aged ≤78 years. A score of ≤5 points for the controlling bladder item of BI along with young recipient age was associated with high caregiver burden that induces depression among caregivers. This approach is useful to identify caregivers with high caregiver burden who are at risk for depression.

## 1. Introduction

The health of family caregivers is crucial for older and disabled people to continue to live at home. Occupational therapists who provide home-based rehabilitation services should support the patients and pay attention to the mental state of family caregivers, reduce the burden of care, and provide necessary support. A large-scale population-based study on 4128 family caregivers of community-dwelling older people under the Long-Term Care Insurance program in Japan reported that 34.2% of the family caregivers were at risk for depression [1]. Furthermore, caregiver depression was associated with high caregiver burden in a large-scale survey in Japan [2] and in a meta-analysis study [3]. Additionally, Arai and Zarit [2] reported that a cutoff score of 13 points in the short version of the Japanese version of the Zarit Caregiver Burden Interview (J-ZBI_8) was associated with depression [4, 5]. Therefore, appropriate support is needed to maintain the J-ZBI_8 score below 13 points to prevent the incidence of depression among caregivers.

Caregiver burden is associated with various elements, including patient factors, caregiver characteristics, and the relationship between patients and caregivers. Patient factors include age [6–8], gender [7], educational level [9, 10], functional disability [7, 11], cognitive impairment [9, 12, 13], and poor activities of daily living (ADL) [10, 12–15]. Occupational therapists are often involved in ADL. Additionally, eating [16], grooming [17, 18], dressing [12, 17, 18], mobility [19, 20], transfer [21], bathing [12, 16, 18], and bowel and bladder management [7, 12, 17, 20, 22–24] have been reported to be associated with caregiver burden. However, to the best of our knowledge, the level of assistance and ADL items that increase the caregiver burden is unknown. Further, the combination of factors associated with high caregiver burden remains elusive.

Therefore, this study was aimed at determining the cutoff values of ADL and the combination of related factors associated with high caregiver burden that induces depression among caregivers. The findings will be useful for occupational therapists to determine ADLs that should be prioritized for intervention based on the caregiver burden. It may also be useful to identify caregivers at risk for depression.

## 2. Materials and Methods

This was a retrospective observational study of 50 pairs of home-based rehabilitation users (patients) and their primary caregivers. Several factors, such as age, gender, disability caused by a disease, and Barthel index (BI) score, were recorded for each patient [25, 26], and the J-ZBI_8 score [2, 3] was recorded for the primary caregivers. Physical or occupational therapists conducted the evaluations. The Research Ethics Committee of the Kita-Fukushima Medical Center (approval no. 88-2) reviewed and approved the study. Considering that our study was retrospective in nature and did not involve intervention, the opt-out method was used instead of obtaining informed consent.

First, we performed correlation analyses and intergroup comparisons to investigate the relationship between the caregiver burden and each of the aforementioned factors. The Spearman rank correlation coefficient (rs) was calculated in the correlation analysis between the J-ZBI_8 scores and each variable. For intergroup comparisons, the subjects were classified into two groups: high-burden and low-burden groups (J-ZBI_8 score ≥ 13 and ≤12, respectively). The Mann–Whitney *U* test and chi-square test were used for intergroup comparisons.

Next, we performed receiver operating characteristic (ROC) curve analysis using the items that showed significant differences in the intergroup comparisons as independent variables and high or low caregiver burden as dependent variables to identify the ADL items and ADL levels associated with high caregiver burden. The Youden index was used to calculate the cutoff value when the area under the ROC curve (AUC) was ≥0.8. Additionally, we performed a decision tree analysis (classification and regression tree) to determine the combination of factors associated with high caregiver burden. The independent variables included the patient's age, gender, disease, and BI, and the dependent variable was high or low caregiver burden. The criterion for the classification of the decision tree was based on the Gini index. To prevent overfitting, cost-complexity pruning (±1 standard error) was performed, and the minimum number of cases in the parent and child nodes was set to 10 and 3, respectively. SPSS Statistics software v25 (IBM Corp., Armonk, NY) was used for all statistical analyses, and the significance level was set at <5%.

## 3. Results

The median J-ZBI_8 score of caregivers was 5.0 (25–75 percentile, 2.0–10.3). Ten caregivers (20%) had a J-ZBI_8 score of ≥13. The correlation analysis showed that the recipient's age (rs = 0.29) and BI feeding (rs = −0.41), transfer (rs = −0.38), grooming (rs = −0.35), toilet (rs = −0.36), bathing (rs = −0.29), mobility (rs = −0.37), dressing (rs = −0.44), controlling bladder (rs = −0.48), controlling bowel (rs = −0.48), and total score (rs = −0.52) were significantly correlated with the J-ZBI_8 scores. Intergroup comparisons showed significant differences in BI transfer (*p* < 0.05), mobility (*p* < 0.05), dressing (*p* < 0.01), controlling bladder (*p* < 0.01), controlling bowel (*p* < 0.05), and total score (*p* < 0.01) (Table 1). The only ADL item with an AUC of ≥0.8 that showed a significant difference between the groups was BI controlling bladder, and the calculated cutoff value associated with high caregiver burden was 5 points (sensitivity: 90%, specificity: 70%).

In the decision tree analysis, the first layer was the BI controlling bladder (≤5 or 10 points) (Figure 1). In the second layer, the recipient's age of ≤78 or ≥79 years was selected in the group in which BI controlling bladder was ≤5 points. High caregiver burden was identified in 85.7% of the caregivers in whom the BI controlling bladder was ≤5 points and the patient was aged ≤78 years. The classification accuracy of the decision tree was 90.0%.

## 4. Discussion

The correlation analysis showed an association between caregiver burden and patient's age and independence level for approximately all ADL items. These findings are similar to those of previous studies [7, 8, 12, 16]. Additionally, the results of the ROC curve and decision tree analyses suggested that among all ADL items, urinary incontinence (controlling bladder) is associated with high levels of caregiver burden (J-ZBI_8 score of ≥13 points) that induces depression among caregivers. A survey by Noelker [27] reported that urinary incontinence is a common issue faced by caregivers, with approximately 53% of older care recipients being incontinent. Tamanini et al. [23] reported that the need to provide care to incontinent older patients may arise without warning, and this care is often provided without adequate caregiver training, which may lead to increased insecurity and anxiety, thus causing physical and mental stress. Further, Tamanini et al. [23] noted that the caregiver has to deal with activities that involve immediate interaction with the patient, such as providing support to patient hygiene, changing diapers or absorbent pads, and exposing themselves to contact with urine and feces. Several studies have reported that urinary incontinence is associated with caregiver burden [7, 12, 17, 22–24], and the present study supports this finding.

The novelty of our study is the finding that a score of ≤5 points on the controlling bladder item of BI is associated with high levels of caregiver burden, which may induce depression among caregivers. Our results suggest that even if urinary incontinence occurs less than once a day, it can be considerably burdensome for caregivers because the functional level indicated by a score of 5 points is “occasional accident” (maximum once per 24 h) [25, 26]. This finding is important for occupational therapists as they support the patients as well as their caregivers. The sensitivity of this cutoff value was 90%, suggesting that it can be used as a simple indicator to identify caregivers who have a high level of caregiver burden that induces depression.

Additionally, according to the decision tree developed in this study, 85.9% of caregivers believed that the caregiver burden was extremely high when the score of the controlling bladder item of BI was <5 points and the patient was aged ≤78 years. It has been reported that the older the patient, the higher the caregiver burden would be [7, 8]; moreover, the results of the correlation analysis in our study also support this finding. However, the decision tree revealed that only when the score of the controlling bladder item of BI was <5 points did the caregiver burden tend to be higher in patients aged ≤78 years than in those aged ≥79 years. Caregiver depression is associated with young [28] as well as old age [29] of the care recipient, and no consensus has been achieved. In this context, our study findings suggest that the association between caregiver depression and the age of the patient varies depending on the presence or absence of urinary incontinence. However, due to the small sample size and limited variables analyzed in our study, future research is necessary to confirm these associations. The decision tree developed in our study may identify caregivers at high risk for depression with even higher accuracy than the single cutoff value of 5 points on the controlling bladder item of BI.

A major limitation of this study is that except ADL, a wide range of factors that are associated with caregiver burden, such as age [9, 11, 13], gender [10, 11, 13, 30], low educational level [11, 30], residing with the care recipient [30], financial stress [30], longer hours of caregiving [13], and health issues [14], were not considered. Because the sample size was insufficient, we were unable to conduct stratified or multivariate analyses. Future studies will require a larger sample size and the use of variables other than ADL to examine the effects of combinations of variables and cutoff values with higher accuracy for detecting caregivers at risk for depression. Additionally, this study was conducted in Japan using the Japanese version of the Zarit Caregiver Burden Interview; therefore, further verification is needed to generalize the results in other countries.

## 5. Conclusions

A score of ≤5 points on the controlling bladder item of BI along with a young recipient age (≤78 years) was associated with high caregiver burden that induces depression among caregivers. This criterion may be used to identify caregivers with high caregiver burden and those at risk for depression.

## Figures and Tables

**Figure 1:** Decision tree associated with high levels of caregiver burden inducing depressive symptoms. BI: Barthel index.

**Table 1:** Characteristics and level of independence in activities of daily living by groups.

	Overall (*N* = 50)	J-ZBI_8 score		*p* value
		≥13 points (*N* = 10)	≤12 points (*N* = 40)	
Age, mean (years)	80.0 (68.8–85.5)	77.0 (70.8–83.5)	80.0 (68.3–87.0)	0.71
Gender, men	23 (46.0)	5 (50.0)	18 (45.0)	1.00
Disease				0.84
Stroke	17 (34.0)	3 (30.0)	14 (35.0)	
Orthopedic diseases	10 (20.0)	3 (30.0)	7 (17.5)	
Neurodegenerative diseases	9 (18.0)	2 (20.0)	7 (17.5)	
Others	14 (28.0)	2 (20.0)	12 (30.0)	
Barthel index				
Feeding	10.0 (10.0–10.0)	7.5 (0.0–10.0)	10.0 (10.0–10.0)	0.07
Transfer	15.0 (10.0–15.0)	10.0 (0.0–15.0)	15.0 (10.0–15.0)	<0.05
Grooming	5.0 (0.0–5.0)	0.0 (0.0–5.0)	5.0 (0.0–5.0)	0.15
Toilet use	10.0 (5.0–10.0)	5.0 (0.0–10.0)	10.0 (5.0–10.0)	0.11
Bathing	0.0 (0.0–0.0)	0.0 (0.0–0.0)	0.0 (0.0–5.0)	0.19
Mobility	5.0 (0.0–15.0)	0.0 (0.0–6.3)	10.0 (0.0–15.0)	<0.05
Stairs	0.0 (0.0–5.0)	0.0 (0.0–5.0)	0.0 (0.0–10.0)	0.38
Dressing	5.0 (0.0–10.0)	2.5 (0.0–5.0)	10.0 (5.0–10.0)	<0.01
Controlling bowel	10.0 (5.0–10.0)	5.0 (0.0–10.0)	10.0 (10.0–10.0)	<0.05
Controlling bladder	10.0 (5.0–10.0)	5.0 (0.0–5.0)	10.0 (5.0–10.0)	<0.01
Total score	70.0 (42.5–85.0)	45.0 (0.0–65.0)	75.0 (51.3–90.0)	<0.01

Median (25–75 percentile) or *n* (%).

## Data Availability

The research data are not shared.
